# The First Occurrence of Angioedema After Discontinuation of Angiotensin-Converting Enzyme Inhibitor

**DOI:** 10.7759/cureus.19553

**Published:** 2021-11-13

**Authors:** Aleesha Kainat, Chen Rong Phang, Noor Ul Ain, Bhawna Agarwal

**Affiliations:** 1 Internal Medicine, University of Pittsburgh Medical Center Mckeesport Hospital, Pittsburgh, USA; 2 Internal Medicine, University of Pittsburgh Medical Center McKeesport Hospital, Pittsburgh, USA

**Keywords:** facial angioedema, bradykinin mediated angioedema, drug-related side effects and adverse reactions, angiotensin-converting enzyme inhibitors, angioedema

## Abstract

Angioedema is one of the dreaded side effects of angiotensin-converting enzyme (ACE) inhibitors. It has been well established in the literature and the timing of onset is variable from months to years after initiation of therapy. Patients remain at risk of recurrence of angioedema even after discontinuation of the drug if they developed it once while on the drug. While only recurrences of ACE inhibitor-induced angioedema are described in the literature, our patient did not develop angioedema while being on the drug and had the first occurrence of angioedema one month after the medication was discontinued. We argue that since our patient did report an ACE inhibitor-related dry cough, this case emphasizes the strength of the relation between the two common side effects of the ACE inhibitors. This favors that among the risk factors that predispose individuals to develop angioedema, ACE inhibitor-associated cough is a major one. Although the mechanism of ACE inhibitor-related cough is poorly understood, bradykinin seems to be the common culprit mediator for these two side effects. Hence, clinicians need to be aware of this potential threat and be cautioned when they witness an ACE inhibitor-related cough.

## Introduction

Angiotensin-converting enzyme (ACE) inhibitors have been well established for their association with angioedema. Another notorious side effect of the ACE inhibitors is dry cough and is manifested in up to 5%-20% of patients [1]. In contrast to other causes of angioedema, which are histamine-related or familial (C1-esterase deficiency), angioedema related to ACE inhibitors is mediated by bradykinin. The mechanism of ACE inhibitor-induced cough is poorly understood but the role of bradykinin has been established [2]. Little is studied about the strength of the relation between these two common side effects [3]. However, bradykinin seems to be the common mediator. Due to the nuisance of dry cough, patients often demand a switch to alternative options, leading to the discontinuation of drugs in such patients [4]. It is however still plausible that patients who manifest a hypersensitivity to ACE inhibitors and develop cough are more likely to develop other reactions as well. Since the timing of onset of both side effects varies from days to years after treatment initiation [5], it is unlikely to predict when a person will manifest the reaction. According to a study, the risk of angioedema persists even after discontinuation of the drug, mostly being recurrences in individuals who manifested angioedema while on the drug [6]. We propose that patients who develop ACE inhibiter-related cough, remain at risk of developing subsequent angioedema even after the drug was discontinued. We present an unusual case of the first occurrence of angioedema one month after discontinuation of ACE inhibitor in a patient due to ACE inhibitor-related dry cough.

## Case presentation

A 60-year-old African American female with a past medical history of hypertension, chronic obstructive pulmonary disease (COPD), hyperlipidemia, sickle cell trait, class III obesity, presented to the hospital with shortness of breath two days ago, associated with a progressively worsening tongue and neck swelling that developed for five days. She was referred to the emergency room from her Primary Care Physician (PCP) office for high clinical suspicion of angioedema. Earlier that day the patient had presented to her PCP office with a progressively worsening, asymmetric (right greater than left) tongue swelling for five days. The tongue swelling had disrupted the patient's sleep and made it difficult for her to swallow solid food. She also endorsed associated painful neck swelling and shortness of breath. She did not notice any rash on her body and denied itching. She also reported having a dry cough for two months, which was persistent despite trying all cough remedies. Her home lisinopril was discontinued four weeks ago with some improvement of cough. She had previously tolerated ACE inhibitor for months without any issue. Upon arrival at the hospital, on physical examination, her vital signs included a temperature of 37.1ºC, blood pressure of 164/89 mmHg, heart rate of 102 beats per minute, respiratory rate of 22 breaths per minute, and oxygen saturation of 93% on room air. She was alert and oriented, speech and voice with wet quality, without stridor, head and neck exam was significant for lower lip swelling, diffuse neck swelling with tenderness, palpable cervical, and retro auricular lymph nodes. A heart exam revealed regular rate and rhythm. Lung examination was notable for decreased air entry bilaterally without any added sounds. Skin exam was without evidence of any erythema, swelling, or rash. The remainder of the examination was unremarkable. Her initial lab work including a comprehensive metabolic panel and complete blood count were within normal limits. Her erythrocyte sedimentation rate was elevated at 59 mm/hr. An initial chest x-ray and x-ray of the soft tissues of the neck were unremarkable. A clinical diagnosis of angioedema related to either ACE inhibitor use or other etiology was made. The patient immediately received steroids, histamine 2 (H2) receptor blockers, Icatibant, and fresh frozen plasma. The patient was evaluated by an otolaryngologist with transnasal flexible fiberoptic laryngoscopy (FFL), which revealed symmetric bilateral watery edema on the lateral edges of the lingual surface of epiglottis without evidence of laryngeal involvement. She was transferred to the Intensive care unit for closer monitoring and anticipated intubation. Further lab testing revealed normal C-1 esterase levels, complement C3 levels, complement C4 levels, and C-reactive protein. The patient’s symptoms persisted on the next day and a repeat FFL evaluation remained unchanged from prior. A computed tomography scan with intravenous contrast of the soft tissues of the neck was obtained which revealed an unremarkable exam of pharyngeal mucosal spaces, larynx, and neck spaces. She was started on antihistamines, H2 receptor blockers, and steroids. The patient received a total five-day course of steroids and had resolution of swelling without requiring intubation. In the absence of associated itching, hives, and normal C-1esterase levels; bradykinin mediated angioedema in the setting of prior ACE inhibitor use was deemed the cause of her angioedema. ACE inhibitor-induced angioedema was permanently added to the list of her allergies. She was transferred to a regular medicine floor within three days and discharged home after a seven-day hospital course with an outpatient follow-up with PCP.

## Discussion

ACE inhibitors are first-line drugs to treat hypertension and are widely prescribed in the United States of America [7]. Angioedema is one of the dreaded side effects of this medication with an incidence of 0.1-0.7 among its recipients [5]. Angioedema is defined as swelling caused by the extravasation of plasma into the surrounding interstitium due to a break in vascular integrity [8]. It most commonly affects the tongue, face, upper airway for instance pharynx, larynx, and subglottic area [9], visceral involvement has also been established [10]. ACE inhibitor-associated angioedema is peculiar as it is not gravity-dependent, and patients do not develop swelling of their feet. The causes of angioedema are broadly categorized into three different classes: mast cell activation (histamine-mediated), bradykinin mediated, or familial (C1 esterase deficiency). The mechanism of ACE inhibitor-related angioedema is thought mainly to be due to elevated bradykinin levels [11]. Unlike histamine-mediated, bradykinin-mediated angioedema does not have associated urticaria [12]. ACE is also known as kinase II enzyme is primarily responsible for the degradation of bradykinin. ACE inhibitors block the kinase II enzyme and hence leading to its impaired metabolism. Bradykinin causes increased release of nitric oxide and prostaglandins. This leads to vasodilation, increased permeability of post-capillary venules, and extravasation of plasma into surrounding submucosal tissue. The timing of onset of ACE inhibitors related angioedema is variable with cases reported within days to years after medication initiation [5]. Recurrence of angioedema even after discontinuation of the drug was also reported in a retrospective study [6]. The symptom spectrum of angioedema ranges from mild swelling to acute respiratory distress in cases of laryngeal involvement. The mainstay of treatment typically involves airway management in cases where edema involves the mouth or throat. Frequent airway assessment should be performed until resolution of swelling is ensured. In any case of airway compromise, equipment, and trained medical personnel should be readily available to proceed with intubation and mechanical ventilation. ACE inhibitors should be discontinued and all drugs from this class should be strictly avoided in the future. Other medical therapies that are frequently used for treatment, are without proper evidence. Fresh frozen plasma which contains the enzyme ACE is often administered (as in our patient) and is believed to degrade the high levels of bradykinin, and resolution of swelling within two to four hours [13]. Icatibant is a synthetic bradykinin B2-receptor antagonist approved for use in acute attacks of hereditary angioedema (HAE). It is often used for ACE inhibitor-induced angioedema with some benefit as manifested in a randomized controlled trial [14], however, expert consensus does not favor its use. Ecallantide, also approved for HAE attacks, works by inhibiting plasma kallikrein and blocks the conversion of high molecular kininogen to bradykinin. Its’ use remains questionable in ACE inhibitor-induced angioedema [15] because ACE inhibitor-induced angioedema is due to decreased degradation of bradykinin rather than overproduction. Tranexamic acid has been studied as initial therapy with some improvement in angioedema [16]. Purified C1 inhibitor concentrate, which works by inhibiting kallikrein, has shown some promise in a few case reports [17,18] if given within hours of symptom onset. Similar to a bradykinin-mediated pathway for ACE inhibitor-induced angioedema, the proposed mechanism for ACE inhibitor-associated cough is also thought to be due to increased bradykinin among other mediators including thromboxane, substance P, and others. [2] Furthermore, ACE inhibitor-related cough was established as an independent strong risk factor for ACE inhibitor-associated angioedema [3]. We propose that a patient who develops an ACE inhibitor-related cough shows a propensity to develop angioedema later and should be monitored even after drug discontinuation. Our case is unique as the patient developed the first episode of angioedema 30 days after discontinuation of the ACE inhibitor. Due to the variable presentations of angioedema that have been reported, it is not implausible to have the first occurrence of angioedema after discontinuation of the medication in a patient who earlier manifested ACE inhibitor-related cough. Proper patient education is mandatory before they are initiated on these medications and should be constantly evaluated for any concerning signs or symptoms while they are on ACE inhibitors. Clinicians should have a lower threshold to offer urgent medical intervention in case of suspected face or neck swelling even after discontinuation of ACE inhibitors.

## Conclusions

ACE inhibitor-related angioedema has an unpredictable course of the presentation, and a recurrence after discontinuation of the drug is also studied. We argue that in a patient manifesting early and benign side effects of the medication such as dry cough, there is a higher propensity to develop subsequent angioedema. Such patients should be monitored for ACE inhibitor-related angioedema and warned about the potentially fatal condition even after discontinuation of the drug. However, given the proven benefits of ACE inhibitors in hypertension and heart failure, this should not deter physicians from prescribing this drug. Proper patient education and a timely clinical diagnosis in such patients are crucial to preventing adverse outcomes.
